# The prognostic potential and carcinogenesis of long non-coding RNA TUG1 in human cholangiocarcinoma

This article has been retracted.

**DOI:** 10.18632/oncotarget.19502

**Published:** 2017-07-22

**Authors:** Yi Xu, Kaiming Leng, Zhenglong Li, Fumin Zhang, Xiangyu Zhong, Pengcheng Kang, Xingming Jiang, Yunfu Cui

**Affiliations:** ^1^ Department of Hepatopancreatobiliary Surgery, Second Affiliated Hospital of Harbin Medical University, Harbin, China; ^2^ Department of The Key Laboratory of Myocardial Ischemia, Harbin Medical University, Ministry of Education, Harbin, China

**Keywords:** cholangiocarcinoma, lncRNA, TUG1, prognosis, EMT

## Abstract

Cholangiocarcinoma (CCA) is a fatal disease with increasing worldwide incidence and is characterized by poor prognosis due to its poor response to conventional chemotherapy or radiotherapy. Long non-coding RNAs (lncRNAs) play key roles in multiple human cancers, including CCA. Cancer progression related lncRNA taurine-up-regulated gene 1 (TUG1) was reported to be involved in human carcinomas. However, the impact of TUG1 in CCA is unclear. The aim of this study was to explore the expression pattern of TUG1 and evaluate its clinical significance as well as prognostic potential in CCA. In addition, the functional roles of TUG1 including cell proliferation, apoptosis, migration, invasion and epithelial-mesenchymal transition (EMT), were evaluated after TUG1 silencing. Our data demonstrated up-regulation of TUG1 in both CCA tissues and cell lines. Moreover, overexpression of TUG1 is linked to tumor size (*p*=0.005), TNM stage (*p*=0.013), postoperative recurrence (*p*=0.036) and overall survival (*p*=0.010) of CCA patients. Furthermore, down-regulation of TUG1 following RNA silencing reduced cell growth and increased apoptosis in CCA cells. Additionally, TUG1 suppression inhibited metastasis potential *in vitro* by reversing EMT. Overall, our results suggest that TUG1 may be a rational CCA-related prognostic factor and therapeutic target.

## INTRODUCTION

Cholangiocarcinoma (CCA) is a carcinoma derived from neoplastic transformation of biliary epithelial cells located in the intrahepatic and extrahepatic bile ducts. It is the second most common primary liver malignant tumor after hepatocellular carcinoma (HCC) and the most common biliary tract malignancy worldwide [1, 2]. Depending on its anatomic location, CCA is generally classified into three types, intrahepatic cholangiocarcinoma (ICC), hilar cholangiocarcinoma and extrahepatic cholangiocarcinoma (ECC) [3]. CCA is a deadly carcinoma with poor prognosis worldwide and is characterized by its resistance to conventional chemotherapy and radiotherapy, in addition to a lack of available methods for early diagnosis and treatment [4, 5]. Unfortunately, the majority of patients diagnosed with CCA present are at an advanced stage [6]. Surgical resection, along with liver transplantation, is still the most powerful therapy to cure CCA and leads to long-term survival. However, surgery is only possible in a significant minority of patients who present at an early stage and the 5-year survival rate of CCA is only 10% [7]. Recent molecular biology studies on the pathogenesis of CCA may provide valid treatment strategies and improve the prognosis of CCA [8]. However, the precise mechanism associated with malignant pathogenesis and progression of CCA remains unclear.

Long non-coding RNAs (lncRNAs) have drawn much attention because of their diagnostic, prognostic, and predictive potential. LncRNAs, a new class and major member of the ncRNA family, are composed of at least 200 nucleotides and have limited or no protein-coding potential [9–11]. However, lncRNAs play crucial roles in the regulation of multiple biological processes related to cancer progression, tumor growth and drug resistance [12–14]. Furthermore, evidence suggests that aberrant lncRNA expression can function as a tumor suppressor [15] or oncogene [16]. For example, lncRNA H19 promotes glioma progression by targeting miR-675 [17]. In addition, the decreased expression of miR-125a-5p after lncRNA HOTAIR knockdown increases cell apoptosis by activating caspase-2 [18].

Taurine-up-regulated gene 1 (TUG1), a 7.1-kb lncRNA, was originally identified as a transcript up-regulated by taurine treatment in developing newborn mice retinal cells. Inhibition of TUG1 expression can prevent proliferation of retinal cells, which suggests a moderating effect of TUG1 on cell growth and its participation in human tumor progression [19]. Several recent studies have confirmed TUG1 overexpression in various types of human tumors and an involvement in carcinogenesis and cancer progression. It has been reported that TUG1 is up-regulated in esophageal squamous cell carcinoma, colorectal cancer, hepatocellular carcinoma, gastric cancer, bladder cancer and hepatoblastoma and therefore promotes tumor progression [20–25]. On the other hand, TUG1 seems to be silenced in glioma and non-small cell lung cancer (NSCLC) [26–29], and thus, TUG1 may suppress the growth of some types of tumors.

Although TUG1 has been shown to have imperative functions in an increasing number of carcinomas, little is known about the expression pattern and exact role of TUG1 in human CCA. In our present study, we aimed to explore the relative expression levels of TUG1 in CCA tissues and corresponding adjacent normal tissues, and assessed the association of TUG1 with clinicopathologic features. In addition, we analyzed CCA cell growth, apoptosis, migration, invasion and epithelial-mesenchymal transition (EMT) after knockdown of TUG1 *in vitro*. This is the first study to reveal the functional role of TUG1 in CCA.

## RESULTS

### TUG1 is upregulated in CCA tissues and cell lines

To explore the expression levels of TUG1 in CCA, qRT-PCR experiments were performed on 51 pairs of CCA tissues as well as diverse CCA cell lines including KMBC, HCCC-9810, HuCCT1, CCLP-1, Huh-28, QBC939 and RBE. Additionally, we examined HIBEC cells as a control. qRT-PCR revealed that TUG1 mRNA levels were up-regulated in CCA tissue samples compared to paired non-tumor tissue with an average fold change of 3.00 (*p*=0.003; Figure 1A). In addition, the majority of cell lines showed substantially higher levels of TUG1 expression compared to HIBEC cells, indicating that TUG1 might be involved in tumorigenesis and progression of CCA (Huh28, *p*=0.038; KMBC, *p*=0.033; HuCCT1, *p*=0.003; QBC939, *p*<0.001; RBE, *p*<0.001; Figure 1B).

**Figure 1:** TUG1 is upregulated in both CCA tissues and cell lines, and overexpressed TUG1 decreased overall survival in patients with CCA **(A)** TUG1 expression levels in CCA tissue samples and adjacent normal tissues; **(B)** TUG1 expression levels in CCA cell lines and HIBEC; **(C)** Kaplan–Meier survival analysis applied based on postoperative survival time and TUG1 expression. *p<0.05, **p<0.01, ***p<0.001.

### TUG1 overexpression is correlated with poor prognosis in CCA patients

To evaluate whether TUG1 may act as a potential diagnostic biomarker for CCA patients, the association between TUG1 and clinicopathological parameters were evaluated (Table 1). Notably, tumor size (*p*=0.005), TNM stage (*p*=0.013) and postoperative recurrence (*p*=0.036) correlated significantly with up-regulated TUG1 expression. However, patients’ gender, age, lymph node invasion and other parameters were not associated with TUG1. Furthermore, Kaplan–Meier survival analysis and the log-rank test applied based on postoperative survival time and TUG1 expression clearly showed that TUG1 expression was associated with a reduced overall survival time of patients after surgery (*p*=0.010; Figure 1C).

**Table 1:** Association between TUG1 expression and clinicopathological parameters of CCA

Clinicopathological features	No. of patients (n)	TUG1 expression		*p*-value
		High (n)	Low (n)	
Gender				
Male	25	14	11	0.573
Female	26	17	9	
Age				
<60	27	17	10	0.780
≥60	24	14	10	
Tumor site				
Intrahepatic	11	5	6	0.406
Perihilar	20	12	8	
Distal	20	14	6	
Tumor size				
<3	28	12	16	**0.005**
≥3	23	19	4	
Lymph node invasion				
Present	28	18	10	0.774
Absent	23	13	10	
Vascular invasion				
Positive	14	11	3	0.198
Negative	37	20	17	
TNM stage				
I-II	15	5	10	**0.013**
III-IV	36	26	10	
Differentiation grade				
Well/moderately	16	7	9	0.126
Poorly/undifferentiated	35	24	11	
Postoperative recurrence				
Present	41	28	13	**0.036**
Absent	10	3	7	
Serum CEA level				
>5 ng/ml	30	17	13	0.566
≤5 ng/ml	21	14	7	
Serum CA19-9 level				
>37 U/ml	34	19	15	0.373
≤37 U/ml	17	12	5	
HBV infection				
Positive	22	12	10	0.564
Negative	29	19	10	

### TUG1 depletion retarded cell proliferation

To shed light on the *in vitro* functional roles of TUG1 in CCA, four specific RNA interference constructs against TUG1 and a negative control (si-NC) were designed for transfection into QBC939 and RBE cell lines as they express the highest levels of TUG1. We tested transfection efficiency by inverted fluorescence microscopy and calculated the percentage of cells expressing green fluorescent protein (Figure 2A). Additionally, flow cytometry results indicated that the transfection efficiency of the lipofectamine 3000 and si-TUG1/si-NC mixture reached 70%–90% in the two selected cell lines (Figure 2B). Moreover, qRT-PCR analysis revealed that the levels of TUG1 expression in selected cell lines were markedly silenced as shown in Figure 2C. Si-TUG1-2 and -3 were the most effective siRNAs targeting TUG1 compared to scrambled siRNA, and therefore were used in subsequent experiments. CCK-8 and Ki67 assays showed that QBC939 and RBE cell growth was restrained in TUG1 depleted groups (Figure 2D and 2E). Consist with these data, after transfection with si-TUG1-2 or si-TUG1-3, clonogenic ability was remarkedly weakened as shown by the colony formation assay (Figure 2F). Moreover, PCNA was down-regulated after knockdown of TUG1 proved by Western blot assay (Figure 2G).

**Figure 2:** Transfection and knockdown efficiency of TUG1-specific siRNA and TUG1 depletion retarded cell proliferation and colony formation in CCA cells **(A)** CCA cells (QBC939 and RBE) under light microscope and fluorescence microscope after transfection (×100). **(B)** Transfection efficiency of CCA cells (QBC939 and RBE) was detected by flow cytometry. **(C)** CCA cells (QBC939 and RBE) were transfected with si-RNA specifically targeting TUG1 or si-NC, and siRNA-depletion efficiency was examined by real-time PCR. **(D)** The proliferation of CCA cells (QBC939 and RBE) after transfection was measured by CCK-8 proliferation assay. **(E)** The proliferation of CCA cells (QBC939 and RBE) after transfection was measured by Ki67 immunofluorescence assay. **(F)** The colony formation capacity of CCA cells (QBC939 and RBE) after transfection was measured by clonogenic assay. **(G)** The protein level of PCNA in CCA cells (QBC939 and RBE) after transfection was measured by Western blot assay. *p<0.05, **p<0.01, ***p<0.001.

### The role of si-TUG1 in promoting CCA cell apoptosis

In order to investigate the potential impact of TUG1 on apoptosis of CCA cells, flow cytometry analysis, AO/EB double fluorescence staining and TUNEL assay were conducted. A multitude of cells transfected with si-NC were alive and did not stain positive for Annexin-V and PI in both QBC939 and RBE cells, whereas in the si-TUG1 counterpart groups, early and late apoptotic cells increased dramatically (Figure 3A). Subsequent AO/EB and TUNEL staining assays showed similar results (Figure 3B and 3C). It has been reported that down-regulation of TUG1 induced cell apoptosis by stimulating the expression of caspase-3 and caspase-9 in human breast cancer [30]. Similarly, relative activities of caspase-3 and -9 were significantly increased in si-TUG1 treatment groups compared to si-NC group (Figure 4A). The Western blot results demonstrated that silenced TUG1 activated Bax protein expression and restrained the protein level of Bcl-2 compared to negative control group (Figure 4B).

**Figure 3:** Silencing of TUG1 induced apoptosis in CCA cells **(A)** The apoptosis of CCA cells (QBC939 and RBE) after transfection was evaluated by flow cytometry. **(B)** The apoptosis of CCA cells (QBC939 and RBE) after transfection was evaluated by AO/EB double fluorescence staining assay (×200). **(C)** The apoptosis of CCA cells (QBC939 and RBE) after transfection was evaluated by TUNEL staining assay. *p<0.05, **p<0.01.

**Figure 4:** TUG1 depletion facilitated apoptosis by activating caspase-3, -9 and Bax expression, and repressing Bcl-2 expression in CCA cells **(A)** Relative expression of caspase-3 and -9 of CCA cells (QBC939 and RBE) after transfection was read by microplate reader. **(B)** The protein levels of Bax and Bcl-2 in CCA cells (QBC939 and RBE) after transfection were detected by Western blot assay. *p<0.05, **p<0.01.

### Knockdown of TUG1 inhibited CCA cell metastasis *in vitro*

To evaluate the extent of TUG1 function in other aspects of CCA, such as migration and invasion, a wound healing assay and Transwell assay were conducted in QBC939 and RBE cells transfected with si-NC or selected siRNAs specifically targeting TUG1. Interestingly, TUG1 depletion leads to prolonged healing times compared with si-NC groups (Figure 5A). Furthermore, the migratory ability as well as invasion potential of selected cells obviously decreased due to TUG1 depletion (Figure 5B and 5C). The above results demonstrated that the down-regulation of TUG1 greatly suppressed RBE and QBC939 cell metastasis *in vitro*.

**Figure 5:** Knockdown of TUG1 inhibited cell migration and invasion potential in CCA cells **(A)** The migration of CCA cells (QBC939 and RBE) after transfection was examined by wound healing assay (×50). **(B)** The migration of CCA cells (QBC939 and RBE) after transfection was examined by Transwell migration assay (×200). **(C)** The invasion of CCA cells (QBC939 and RBE) after transfection was examined by Transwell invasion assay (×200). *p<0.05, **p<0.01.

### Silenced TUG1 reversed EMT in CCA cells

EMT is closely correlated with cell invasion capacity. Therefore, to assess the relationship between dysregulation of TUG1 and EMT, EMT markers including E-cadherin, N-cadherin and Vimentin were analyzed by Western blot. The results shown in Figure 6A and 6B demonstrated that the protein expression level of E-cadherin was significantly increased, while N-cadherin and Vimentin were lost in QBC939 and RBE cells when TUG1 was silenced. These data implied that the down-regulation of TUG1 reversed EMT in CCA cells.

**Figure 6:** Silenced TUG1 reversed EMT in CCA cells **(A)** The expression levels of EMT-related proteins in QBC939 cells after transfection were determined by Western blot assay. **(B)** The expression levels of EMT-related proteins in RBE cells after transfection were determined by Western blot assay. *p<0.05, **p<0.01.

## DISCUSSION

CCA remains one of the most lethal malignancies among people despite great efforts to reverse this situation. For this reason, it is urgent to identify novel biomarkers to improve the early diagnostic rate and to explore therapeutic targets for CCA patients. LncRNAs were mistaken for useless byproducts of transcription for a long time. However, during the past decade, they were proven to be imperative elements in cell biology and human diseases, especially for various carcinomas. For example, HOTAIR, POU3F3, 91H, ZFAS1 and many other lncRNAs were shown to have multiple fundamental roles in several types of carcinomas [31–34]. To date, several CCA-associated lncRNAs have been recognized. For instance, lncRNA H19 and HULC promote cell migration and invasion using a ceRNA method under oxidative stress [35].

Recently, increasing evidence has indicated that the newly identified lncRNA molecule TUG1 plays crucial roles in tumorigenesis and in the progression of certain types of carcinomas [36] and these data have provided new insights into CCA. Aberrant upregulated TUG1 has been detected in various types of carcinomas, such as osteosarcoma, ovarian cancer, colon cancer, bladder carcinoma, esophageal squamous cell cancer and kidney cancer [37–42]. In bladder cancer, TUG1 suppressed the expression of miR-145 and there was a mutual suppression between TUG1 and miR-145. Besides, ZEB2 functioned as a downstream target of miR-145. Thus, TUG1 exerted an oncogene via miR-145/ZEB2 axis [40]. Huang et al. demonstrated that TUG1 was activated by the nuclear transcription factor SP1 in HCC, and upregulation of TUG1 could inhibit the tumor-suppressor gene Kruppel-like factor 2 (KLF2) via binding to polycomb repressive complex 2 (PRC2) and recruiting it to KLF2 promoter region [22]. Interestingly, TUG1 expression in glioma, along with NSCLC was found to be down-regulated and acted as a tumor suppressor [26–29]. Tissue-specific expression is ubiquitous and might explain this phenomenon [43]. In agreement with all of the digestive system neoplasms studied to date, the results of our investigation verified that TUG1 was higher in CCA tissue samples and CCA cell lines compared with corresponding healthy tissue samples and HIBEC cells, respectively. Additionally, high expression of TUG1 was closely associated with tumor size, TNM stage, postoperative relapse and overall survival of CCA patients. Therefore, lncRNA TUG1 may serve as a potential prognostic indicator for CCA.

Proliferation is one of the most basic characteristics of cancer. Herein, CCK-8 proliferation assay, Ki67 immunofluorescent staining and colony formation assay were performed to evaluate the proliferative activity of CCA. PCNA is widely known as an imperative factor in the metabolism of nucleic acid and mainly functioned in DNA replication, DNA repair, chromatin assembly and RNA transcription [44]. In our study, CCA cell proliferation was remarkedly inhibited along with the loss of PCNA and Ki67 followed by silencing of TUG1, indicating that TUG1 promotes tumor development and progression in CCA.

Apoptosis is an effective pathway to eliminate unnecessary cells. During the past decades, 14 mammalian caspases were identified. Among these, caspase-3 (effector caspase) and caspase-9 (initiator caspase) play key roles in the process of cell apoptosis. Bcl-2 family proteins function as central regulators of cell life and death. Apoptosis signaling can be activated by receptor-mediated pathway and mitochondrial pathway [45]. Both of the pathways are associated with the activation of caspase-3, caspase-9, Bax and Bcl-2 [46]. In the present study, down-regulated TUG1 induced cell apoptosis by activating the expression of caspase-3, -9 and Bax, as well as suppressing Bcl-2 expression. The results suggested that Bcl-2/caspase-3 pathway might play key roles in mediating apoptosis induced by downregulation of TUG1.

EMT, which is characterized by lack of intercellular contacts, increasing components of the contractile cytoskeleton, drives the initiation of metastasis [47, 48]. Conversely, a reverse of EMT is essential for migrating cells to colonize a secondary site. EMT markers, such as E-cadherin and Claudins are down-regulated, whereas non-epithelial markers, especially N-cadherin, Vimentin and Fibronectin are over-expressed in the process of EMT. It has been reported that a switch between E-cadherin and N-cadherin is the key step of invasiveness alteration in CCA [49]. Besides, lncRNAs are emerging as potent regulators of tumor metastasis and EMT [50, 51]. Therefore, a Western blot assay was carried out and revealed that silenced TUG1 could impair migratory and invasive potential of QBC939 and RBE cells by reversing EMT progress. These findings demonstrated that cell metastasis of CCA determined by EMT-related gene expression could be regulated by TUG1 silencing.

In conclusion, our findings provide the first depiction of the biological function of lncRNA TUG1 in CCA. However, further studies are needed to unravel the precise mechanism behind the altered expression of TUG1 in CCA. Collectively, we showed that TUG1 is an important prognostic factor for CCA patients and significantly contributes to CCA progression. These results may provide a strategy and facilitate the exploration of TUG1 directed diagnostics and therapeutics against CCA.

## MATERIALS AND METHODS

### Patients and tissue samples

Fifty-one CCA patients who underwent radical surgical procedures at the Second Affiliated Hospital of Harbin Medical University from 2010 to 2012 were enrolled in the study. All patients gave their written informed consent approved by the Ethics Review Committees of Harbin Medical University. In addition, no patients underwent preoperative anti-cancer therapy. After surgery, fresh tissue specimens were collected and frozen in liquid nitrogen to avoid RNA degradation.

### Cell lines and culture

HCCC-9810 and RBE were commercially obtained from the Cell Bank of Chinese Academy of Sciences (Shanghai, China). Human intrahepatic biliary epithelial cells (HIBEC), and CCA cell lines including QBC939, Huh-28, HuCCT1, KMBC and CCLP-1 were preserved in our laboratory. Cells were cultured in dulbecco's modified eagle medium (DMEM) or RPMI-1640 containing 10% fetal bovine serum (FBS) (Invitrogen Life Technologies, USA) in a 37°C humidified atmosphere at 5% CO_2_. All cell lines were passaged for no more than six months.

### RNA extraction and qRT-PCR

Total RNA from samples or cells were extracted by TRIzol reagent (Invitrogen, Waltham, USA) following the manufacturer’s recommendations and converted to cDNA using Transcriptor First Strand cDNA Synthesis Kit (Roche, Germany). qRT-PCR was performed with FastStart Universal SYBR Green Master (Roche, Germany) in a BIO-RAD C1000 Thermal Cycler. GAPDH served as an endogenous control. The following primer sets for TUG1 or GAPDH were used for real-time PCR: TUG1 Forward, 5′- TAGCAGTTCCCCAATCCTTG -3′ Reverse, 5′- CACAAATTCCCATCATTCCC -3′; GAPDH Forward, 5′- GGGAGCCAAAAGGGTCAT -3′ Reverse, 5′- GAGTCCTTCCACGATACCAA -3′. Gene expression was calculated by delta-delta CT method.

### siRNAs and transfection

Cells were transfected with either a small interfering RNA targeting TUG1 or the nonspecific scrambled siRNA (GenePharma, Shanghai, China) using Lipofectamine 3000 (Invitrogen) and serum-free medium. Following transfection (6 h), cells were transferred to complete medium with 10% FBS and antibiotics. Fluorescently labeled siRNAs were counted using an inverted fluorescence microscope, flow cytometry was used to examine transfection efficiency, and TUG1 depletion efficiencies were analyzed by real time PCR. The target sequences of si-TUG1 are shown below: si-TUG1-1, sense 5′- CCUCAGAUCUCAUCUAAAUTT -3′ antisense 5′- AUUUAGAUGAGAUCUGAGGTT -3′; si-TUG1-2, sense 5′- GCGAGUCACUCUGUAAUUUTT -3′ antisense 5′- AAAUUACAGAGUGACUCGCTT -3′; si-TUG1-3, sense 5′- GCUUGGCUUCUAUUCU GAAUCCUUU -3′ antisense 5′- AAAGGAUUCAGAAU AGAAGCCAAGC -3′; si-TUG1-4, sense 5′- GGAUAUAGCCAGAGAACAATT -3′ antisense 5′- UUGUUCUCUGGCUAUAUCCTT -3′.

### Proliferation assays

For CCK-8 analysis, QBC939 and RBE cells transfected with TUG1 siRNA or si-NC were transferred into 96-well plates at a concentration of 1500 cells per well. Cell Counting Kit-8 (Dojindo, Tokyo, Japan) was used to assess cell viability. Reagents were added into corresponding wells at each monitored time (0, 24, 48, 72, and 96 h) and the plate was then incubated at 37°C for 1.5 h before absorbance at 450 nm was measured using a microplate reader (Tecan). For the Ki67 immunofluorescence assay, treated cells were planted into 24-well plates on cover glass. Briefly, after fixation with Immunostaining Permeabilization Buffer with Triton X-100 (Beyotime, Beijing, China) and blocked with 5% bovine serum albumin, cells were incubated with anti-Ki67 monoclonal antibody (Abcam, USA) overnight at 4°C. Next, cells were probed with secondary antibody and 4, 6-Diamidino-2-phenylindole (DAPI) (Beyotime, Beijing, China) was applied to color the nuclei. An inverted fluorescent microscope (Leica, Germany) was used to observe and take photographs. For the clonogenic assay, QBC939 and RBE cells were trypsinized into a single-cell suspension and plated in a 3.5-cm dish at a total of 500 cells per well. The cells were maintained in an incubator for approximately 2 weeks until there were visible colonies formation. After fixation with paraformaldehyde and staining with crystal violet (Beyotime, Beijing, China), colonies were counted from three randomly chosen fields.

### Flow cytometry for cell apoptosis

To detect apoptosis, transfected cells were collected and washed twice with cold PBS. The cells were measured by flow cytometry (FACScan; BD Biosciences, USA) after double staining with 5 μl FITC-Annexin V and 5 μl Propidium iodide (PI) using FITC Annexin V Apoptosis Detection Kit (BD, Biosciences, USA) in accordance with the manufacturer’s recommendations. The percentage of apoptotic cells was determined and then compared in each group.

### Acridine orange/ethidium bromide (AO/EB) double fluorescence staining

Cells transfected with si-TUG1 or si-NC in the exponential growth phase were cultured in an incubator of 5% CO_2_ at 37°C, followed by staining with prepared AO/EB mixing solution for 5 min (Solarbio, Beijing, China). AO/EB staining could distinguish live cells from apoptotic cells by their different abilities to penetrate the cell membrane. AO could permeate intact cell membrane and color the nuclei in green fluorescence. Conversely, EB stains DNA with orange fluorescence only when the cell membrane is broken. A fluorescence microscope (Leica, Germany) was used to count and take photographs.

### TdT-mediated dUTP Nick-End Labeling (TUNEL) assay

One Step TUNEL Apoptosis Assay Kit (Beyotime, Beijing, China) was used to detect cell apoptosis. Treated cells were fixed with paraformaldehyde for 30 min. After washing with PBS, cells were incubated with Immunostaining Permeabilization Buffer with Triton X-100 (Beyotime, Beijing, China). Afterwards, cells were treated with 45 μl fluorescent labeled reagent and 5 μl terminal deoxynucleotidyl transferase (TdT) before incubated at 37°C for 60 min. Cells were observed by a fluorescent microscope (Leica, Germany).

### Caspases analysis

Total cell proteins were extracted after 48 h siRNA treatment, and 10 μl protein from each group was incubated with 90 μl of provided reaction buffer and Ac-DEVD-*p*NA (2 mM) in 96-well plates at 37°C for 4 h following the manufacturer’s instructions (Solarbio, Beijing, China). Afterwards, reaction mixtures were detected using a microplate reader at a wavelength of 405 nm and relative activities of caspase-3 and -9 were compared between the si-TUG1 groups and the corresponding si-NC group.

### Scratch wound assay

Transfected cells were seeded as a monolayer in 3.5-cm dishes and cultured to a density of 80%. Then, straight wounds were softly scratched by a sterile 200-μL pipette tip and rinsed three times with phosphate buffer solution (PBS) to clean up cellular debris. Photographs were taken 0 h and 36 h after wound formation.

### Migration and invasion assay

To analyze the degree of migration, QBC939 and RBE cells (5 × 10^4^ cells/well) were detached with serum-free RPMI-1640 and loaded in the upper section of a 24-well transwell unit with 8-μm polycarbonate nucleopore filters (Corning, NY, USA). The lower chamber was filled with 600 μl medium containing 10% FBS. The transwell unit was incubated for 24 h before the cells on the lower surface of the membrane were fixed and stained with crystal violet. Cells from at least five representative fields were analyzed. For the invasion assay, 40 μL Matrigel (BD Biosciences, San Jose, CA, USA) was coated in the top filter of the transwell unit and placed in an incubator at 37°C for 4 h to form a reconstructed basement membrane. The methods used were identical to those applied to the migration assay.

### Western blot analysis

Forty-eight hours post-transfection, QBC939 or RBE cells were digested with trypsin (Beyotime, Beijing, China) and lysed with RIPA lysis buffer (Beyotime, Beijing, China) supplemented with protease inhibitors. Equal amounts of extracted proteins were fractionated by sodium dodecyl sulfate polyacrylamide gel (SDS-PAGE) vertical electrophoresis, followed by transfer onto a 0.45 μm polyvinylidene fluoride (PVDF) membrane (GE Healthcare, Piscataway, NJ, USA). The membrane was blocked with 5% skim milk diluted in Tris-buffered saline containing 0.05% Tween-20 for 1.5 h at room temperature and then probed with primary antibodies to E-cadherin, N-cadherin, Vimentin, PCNA, Bax or Bcl-2 (Abcam, USA) overnight. After washing and incubating with secondary antibody (Cell Signaling Technology, Danvers, USA) for 2 h, BeyoECL Plus Kit (Beyotime, Beijing, China) was used to visualize the blots.

### Statistical analysis

Data were obtained from at least three independent experiments, presented as the mean ± standard deviation (SD), and analyzed using Student’s t test. Fisher’s exact test was used in clinicopathological associations of TUG1 expression. A *p*<0.05 value was considered significant.

## Abbreviations

AO/EB: acridine orange/ethidium bromide
CA19-9: carbohydrate antigen 19-9
CCA: cholangiocarcinoma
CEA: carcino embryonie antigen
DAPI: 4, 6-diamidino-2-phenylindole
DMEM: dulbecco's modified eagle medium
ECC: extrahepatic cholangiocarcinoma
EMT: epithelial-mesenchymal transition
FBS: fetal bovine serum
HCC: hepatocellular carcinoma
HBV: hepatitis B virus
HIBEC: human intrahepatic biliary epithelial cell
ICC: intrahepatic cholangiocarcinoma
KLF2: Kruppel-like factor 2
lncRNA: long non-coding RNA
NSCLC: non-small cell lung cancer
PBS: phosphate buffer solution
PCNA: proliferating cell nuclear antigen
PI: propidium iodide
PVDF: polyvinylidene fluoride
SD: standard deviation
SDS-PAGE: sodium dodecyl sulfate polyacrylamide gel
TdT: terminal deoxynucleotidyl transferase
TUG1: taurine-upregulated gene 1
TUNEL: TdT-mediated dUTP Nick-End Labeling
